The article "Clinical and Epidemiological Interventions for Monkeypox Management in Children: A Systematic Review" was retracted in 2025. Reasons: unreliable results or conclusions; concerns about the data.

# Clinical and Epidemiological Interventions for Monkeypox Management in Children: A Systematic Review

**DOI:** 10.7759/cureus.38521

**Published:** 2023-05-04

**Authors:** Viral Maru, Usama bin Ghaffar, Anurag Rawat, Mohammed Yunus, Akshayraj K Langaliya, Shubhangi Vyas, Dhaval Mehta, Akshaya Ojha

**Affiliations:** 1 Pediatric Dentistry, Government Dental College and Hospital, Mumbai, IND; 2 Basic Sciences, Majmaah University, Al Majmaah, SAU; 3 Interventional Cardiology, Himalayan Institute of Medical Sciences, Dehradun, IND; 4 Pathology, Imam Abdulrahman Bin Faisal University, Dammam, SAU; 5 Conservative Dentistry and Endodontics, AMC Dental College and Hospital, Ahmedabad, IND; 6 Dentistry, AMC Dental College and Hospital, Ahmedabad, IND; 7 Oral Medicine and Radiology, Narsinhbhai Patel Dental College and Hospital, Sankalchand Patel University, Visnagar, IND; 8 Pediatric Dentistry, Private Practice, Jammu, IND

**Keywords:** intervention, management, children, monkey pox, a systematic review

## Abstract

This review aims to compile the available literature on monkeypox, identify risk factors for developing the disease, and recommend effective preventative methods to reduce the number of reported cases and fatalities in children and pregnant women. In seeking out pertinent studies on monkeypox virus in children and pregnant women, we searched the literature using the databases Cochrane Library, Google Scholar, PubMed, EMBASE, Web of Science, and Scopus up to 1st February 2023. This study analyzed data from case studies of monkeypox in children and pregnant women. Clinical data and test findings of monkeypox patients less than 18 years old and pregnant women were analyzed. The Newcastle-Ottawa Scale was used to do the quality evaluation. Our record examination spanned the years 1985 to 2023 and found 17 children and five pregnant female patients treated with monkeypox in various hospitals/community centers. Zaire, Gabon, Chicago, Sierra Leone, Central African Republic, Northern DR Congo, Liberia, Cameroon, the Democratic Republic of the Congo, the United Kingdom, the Netherlands, and Florida all contributed to the 14 studies analyzed. There were no studies identified for meta-analysis of selected case studies of hospitalized children and pregnant women who were diagnosed with monkeypox. The incidence, prevalence, clinical characteristics, diagnosis, management, prevention, vaccinations, infant care, and care for expectant mothers are all discussed in this systematic review of monkeypox in children. Our research findings may provide a foundation for further focused research and the development of related recommendations or guidelines.

## Introduction and background

The current multi-nation epidemic of the monkeypox virus (MPV) has drawn interest from around the world since it has mostly impacted non-endemic places, such as numerous European nations, Canada, the US, and Australia [1]. In children under the age of 10 years, the possibility of MPV's cross-border diffusion and subsequent transmission has risen due to ambiguity surrounding the containment of the epidemic and the danger of transmission at the social level. The MPV is a member of the family Orthopoxviruses and has a DNA double helix [2-4] and is first seen in monkeys; it subsequently was shown to infect other species, including dormice, Gambian pouched rats, tree squirrels, and string squirrels [5]. Infection with the MPV was first detected in a male child in the Democratic Republic of the Congo (DRC, formerly known as Zaire) in 1970 [6], and subsequent cases have mostly occurred in West and Central Africa [7].

The MPV was previously just a problem in Africa, but now that isolated cases have been found in the West, it poses a hazard to humans all across the globe. Human-to-human transmission often occurs by inhalation of contaminated droplets or skin-to-skin contact with an infected person's mucocutaneous sores, making social seclusion and contact monitoring necessary. Higher incidences of MPV have been observed in people in their mid-twenties. The World Health Organization (WHO) documented 15,734 MPV as of 21 July 2022 in 75 nations across five continents, including children. The possibility of a major public health disaster of concern on a global scale is demonstrated by the poxvirus’s unprecedentedly extensive geographic dissemination [8]. 

According to the scant information from prior outbreaks, children may be more susceptible to the disease’s severe manifestations, leading to sepsis, encephalitis, and even death or long-term disability. Additionally, reports recommend that babies delivered to mothers who have MPV while pregnant should be properly monitored in a special care facility. However, because of inadequate epidemiological monitoring and low access to diagnostic techniques in resource-constrained settings, the pediatric population has only been the subject of tiny case series in the literature [9]. As a result, the current investigation was carried out to put forward the first baseline data on the issue for future comparisons. With regard to the epidemiology of MPV in children, prevalence, clinical traits, diagnosis, therapy, prevention, vaccines, newborn care, and care for expecting moms, this research will focus on current developments throughout the assessment. In addition, this evaluation will include recommendations or guidelines from the Centres for Disease Control and Prevention (CDC).

## Review

This is an in-depth analysis of the epidemiology, diagnosis, prevention measures, prevalence projections, vaccinations, and clinical care standards for the MPV epidemic in children. This investigation also includes recommendations for therapy or supportive care for children up to the age of 18 years, pregnant women, and fetuses. The work is listed in the prospective worldwide registry of systematic reviews (PROSPERO) and Preferred Reporting Items for Systematic Reviews and Meta-Analyses Protocol (PRISMA-P) criteria that are used for conducting this systematic review (CRD 42022368898) [10]. Up to 1st February 2023, three authors (MV, GU, and RA) independently examined electronic databases, including Cochrane Library, Google Scholar, PubMed, EMBASE, Web of Science, and Scopus. “Human,” “Monkeypox Virus,” “Epidemiology,” “Child,” “Orthopoxvirus,” “vaccination,” “Preschool Child,” and “Newborn” were the MeSH words or free text terms that were utilized. We looked over the secondary sources in grey literature, including textbooks and major publications. Additionally, every article that was recognized as being relevant had its reference list extensively examined. Only those articles that have full texts available in English were included.

Research question

The present review is intended to address the following research question: Is the MPV responsible for the reported child/fetal fatalities in endemic areas, and if so, what preventative actions should be taken to protect children and pregnant women from this disease? In this systematic analysis, we review details of all patients up to the age of 18 years and pregnant women with positive MPV polymerase chain reaction (PCR) from any anatomical site, such as skin lesions, blood, serology, or culture. We gathered clinical information (such as demographics, disease complications, symptoms and signs upon presentation, and any antiviral medications used) and laboratory findings (including MPV PCR results and routine biochemical tests). Minors, including those under 18 years, and expectant mothers with MPV who received therapy, a placebo, or routine care were studied for clinical data and laboratory results. The pathophysiology, diagnosis, preventative strategies, vaccines, side effects, and clinical characteristics of MPV in minors, including those under 18 years, and expectant mothers are discussed in this article. The use of real-time PCR assays to confirm the infection is discussed in this report, along with information on the diagnostic options for treating MPV in children under the age of 18 and pregnant women. Additionally, the study offers guidelines and suggestions to safeguard the health of fetuses, minors, including those under 18 years, and expectant mothers exposed to the MPV.

Inclusion criteria

The following criteria were used to decide which papers to include in our systematic review: For inclusion of in vitro studies, the following criteria must be met: (1) only studies that evaluated the diagnostic tool and effectiveness of various medications or treatment options for MPV in children and pregnant women; (2) studies that reported data on the cytotoxicity and inhibitory effect of the drug; (3) published case studies. Clinical studies that encompassed the following requirements were taken into account: (1) case-control studies, randomized controlled trials (RCTs), cohort studies, and non-RCTs; (2) studies designed to evaluate various diagnostic tools and treatment options for MPV in children; (3) studies with a major treatment medication that include a control group receiving either conventional care/control or a placebo; (4) performed only on humans; (5) either published or full preprints available.

Exclusion criteria

The following clinical and in vitro research studies were disregarded throughout our systematic review: (1) RCTs with just one treatment; (2) conducted on animal models; (3) completed trials with results that have not been published or full texts of preprints that are not accessible; (4) active, enrolled clinical trials; (5) missing information about intended results (criteria for clinical studies); (6) studies available in languages other than English.

After searching the literature, two authors (YM and LA) individually checked each title and abstract against the qualifying requirements. Each qualifying research’s first author, publication year, study design, outcome measures, treatments (including the type of treatment used), sample size, and key findings were all retrieved. Each author reached a consensus to settle any differences. Two independent authors (VS and MD) used the Newcastle-Ottawa Scale or non-RCTs, case-control studies, and cohort, and the new Cochrane risk of bias tool for randomized controlled trials (ROB-2) for RCTs to evaluate the quality of only the clinical studies that were included in our systematic review [11]. Any disagreements were settled through discussion with the review’s remaining authors.

In this research, a review was conducted on hospitalized children and pregnant women with confirmed MPV. Our record examination spanned the years 1985 to 2023 and found 17 children and five pregnant female patients treated with MPV in various hospitals/community centers (Figure 1).

**Figure 1:** PRISMA flow diagram PRISMA: Preferred Reporting Items for Systematic Reviews and Meta-Analyses Protocol

Zaire, Gabon, Chicago, Sierra Leone, Central African Republic, Northern DR Congo, Liberia, Cameroon, the DRC, the United Kingdom, the Netherlands, and Florida all contributed to the 14 studies analyzed. Using the Newcastle-Ottawa scale, the majority of research received ratings between one and six (Table 1).

**Table 1:** Evaluation of the included studies using the Newcastle-Ottawa scale

Study	Overall star rating
Stagles et al., 1985 [12]	1
Müller et al., 1988 [13]	1
Anderson et al., 2003 [14]	5
Reynolds et al., 2019 [15]	5
Nakoune et al., 2017 [16]	6
Mbala et al., 2017a [17]	4
Eltvedt et al., 2020 [18]	3
Ngbolu et al., 2020 [19]	4
Larway et al., 2021 [20]	6
Gweh et al., 2021 [21]	4
Jarman et al., 2022 [22]	6
Adler et al., 2022 [23]	3
Tutu van Furth et al., 2022 [24]	5
Saunders et al., 2022 [25]	2

We retrieved clinical information, including demographic factors, symptoms, complications of the disease, therapies received, and laboratory test findings. We have described here MPV spread via different channels: family, health care, and travel. In addition, the WHO clinical severity score based on the number of skin lesions was used to define human MPV cases as mild (<25 skin lesions), moderate (25-99 skin lesions), severe (100-250 skin lesions), or fatal (>250 skin lesions) [26].

Analysis of the clinical progression and therapeutic response in children/pregnant women with MPV

Post-mortem examination of a single cutaneous MPV lesion from Patient 1, who passed away after five days of illness, showed that infected epidermal cells contained many orthopoxvirus fragments, as determined by histological and electron microscopic analysis [12]. Patient 2, a nine-month-old girl, ruled out Marburg, yellow fever, Dengue, and Lassa viruses by serological testing. Despite getting antibiotic and quinine medication, the infant died 48 hours after hospitalization. In this instance, post-mortem liver and spleen samples were examined for the presence of MPV [13].

The emergency department transferred a White schoolgirl (Patient 3) to a Midwest hospital. Patient 3 and her family acquired a prairie dog at a Chicago trade meet a month before admission. The prairie dog became unwell and died soon after purchase for unclear reasons. On the fourth day of hospitalization, she was able to eat and drink normally, and the cervical lymph adenopathy continued to diminish. Many lesions fell off throughout the night, and around 80% of them crusted over or were umbilicated [14].

The finding of MPV infection in a toddler of 11 months (Patient 4) reveals the likely reappearance of MPV in Sierra Leone, where it has not been documented for 44 years [15]. In comparison, the first two clinical instances occurred in youngsters aged 5 (Patient 5) and 9 (Patient 6) from a hunting family dwelling in the hamlet of Madigui, about 10 kilometers from the city of Bakouma. The index patient, a nine-year-old child, became ill after hunting and chopping up a mouse identified as Thryonomis and known locally as “cibissi” [16]. The mother, 15-month-old brother (Patient 7), and maternal aunt all had the illness at the same time as the boys. Five non-family members also showed signs of the illness: a hospital nurse, a doctor, a carer who accompanied patients on transport to a medical facility, and two people who drove them there. Children as young as 15 months and as old as five years old, the two younger brothers of the initial case, were among the 10 people who became unwell and were among the seven who required hospitalization [16].

The reported case of Patient 8 exemplifies a number of difficulties associated with the local management of the condition. This includes lacking diagnostic equipment in rural health centers and failure to recognize the disease by health workers. Also, practical hurdles, such as a lack of knowledge on collecting and transferring a sample and staff nervousness about handling infected material, have been seen in other countries and slowed down the diagnosis process [18].

The eight-year-old boy patient, Patient 9, arrived with headache, fever, and rashes. His mother (main suspect) was a farmer who was married to a hunter. She felt better two weeks before her son’s due date while experiencing the same symptoms. There was no proof that the primary case had eaten bush meat, despite the fact that the patient’s husband was a hunter. The mother and her kid have never gone outside of their own region. Both conditions responded well to symptomatic therapy. However, research was unable to identify the infection’s primary source [20].

The West African MPV was detected in Patient 10, a five-year-old Liberian kid from the Tenken Village in Maryland County. In this particular case, the patient had never been exposed to wild animals or ingested any vegetation, nor had they ever traveled or came into contact with a sick person. Three weeks of therapy with analgesics and antibiotics resulted in the patient’s recovery. No clues pointed to a specific source of the illness. The delay was caused by the unavailability of MPV testing facilities in Liberia since samples had to be sent to Atlanta, Georgia, in the United States [21].

During a measles immunization and monitoring effort after an epidemic of measles, Patient 11, a 14-year-old boy with a fever and a rash, was found. This condition resulted from touching a huge forest rat. The diagnosis of MPV was confirmed using PCR. His rash improved after seven days when it crusted, and his fever subsided. Despite the fact that this case was found after a measles vaccination drive, differentiating MPV from chicken pox is sometimes the largest diagnostic obstacle. The diagnostic challenge in this case was exacerbated by the negative whole-blood PCR [22].

Patients 12, 13, and 14 are the first reported cases of MPV in the province of Nord Ubangi. Monkeypox-specific epidemiological features included high fevers, rashes, itching, and stomach discomfort. Each patient was able to leave without additional difficulties after two weeks of symptomatic therapy [19].

Patient 15 was diagnosed with MPV soon after arriving in the United Kingdom from Nigeria. She was infected by her MPV-positive father. After PCR analysis of a lesion swab confirmed the presence of MPV, the youngster was hospitalized. The youngster was treated in the adult HCID unit with pediatric professionals on-site 24 hours a day. Doctors considered treating the child with tecovirimat but ultimately decided against it since the drug is not yet approved for pediatric usage, there is no established dosage for patients weighing less than 13 kg, and the drug has only been used in one case of pediatric vaccinia infection. All lesions were crusted over by day 12 of illness, although MPV DNA was still detectable by PCR in nasopharyngeal swabs taken on day 20 [23].

A male youngster less than 10 years old (Patient 16) arrived at a pediatric emergency department (ER) in Amsterdam, Netherlands, at the end of June 2022. He had no relevant medical history. He was immunized in accordance with the Dutch national immunization program and contracted chicken pox at age 5. The levels of leukocytes, thrombocytes, and hemoglobin were all within the normal range. The patient’s DNA was located within the clade 3 lineages B.1 but was not directly linked to other strains from the Amsterdam area using whole genome sequencing [24]. On the other side, Patient 17, a two-month-old newborn, was found positive for Orthopoxvirus DNA and Clade II MPV DNA 10 days after the rash’s development [25].

Three of four pregnant women (Patients 18, 19, 20, and 21) diagnosed with MPV infection lost their fetuses. As the miscarriage babies were not examined, there was no indication of fetal contamination in the two spontaneous abortions that occurred during the first trimester of pregnancy. Complications from a clinically apparent maternal MPV infection likely led to the intrauterine mortality of a fetus in a lady who was 18 weeks pregnant with moderately severe MPV. The maternal MPV load rose rapidly and abruptly from 102 to 106 genome copies/mL from day 21 to 23 after the illness, which coincided with stopping of the fetal movement. Increased vascular permeability and extensive hepatic involvement in the fetus’s hepatomegaly and peritoneal effusion (hydrops fetalis) were likely the results of MPV-induced cellular damage [17]. A summary of the clinical progression and therapeutic response of MPV in children and pregnant women is provided in Tables 2, 3, respectively.

**Table 2:** Analysis of the clinical progression and therapeutic response of monkeypox virus in children MPV: Monkeypox virus; qPCR: quantitative polymerase chain reaction

Patient number	1 [12]	2 [13]	3 [14]	4 [15]	5 [16]	6 [6]	7 [16]	8 [18]	9 [20]	10 [21]	11 [22]	12 [19]	13 [19]	14 [19]	15 [23]	16 [24]	17 [25]
Year of infection	1985	1987	2003	2014	2015	2015	2015	2016	2017	2017	2019	2019	2019	2019	2021	2022	2022
Age	2	9-month	Not specified	11-month	5	9	15-month	4	8	5	14	13	7	7	<2	10	<2 months
Sex	Male	Female	Female	Male	Male	Male	Male	Male	Male	Male	Male	Male	Male	Male	Female	Male	-
Transmission cause	-	-	Prairie dog	Parents consume meat from wild animals	From infected brother	Contact with rodent known locally as “cibissi”	Breastfeeding	-	Father is a hunter	-	Contact with a giant forest rat	Tapper of rats and squirrels	-	-	-	-	-
Mode of transmission	Unknown	Unknown	Direct	Direct	Familial	Direct	Familial	Unknown	Familial	Unknown	Direct	Direct	Familial	Unknown	Travel	Travel	Unknown
Country of acquisition	Zaire	Gabon	Chicago	Sierra Leone	Central African Republic	Central African Republic	Central African Republic	Northern Democratic Republic of the Congo	Liberia	Liberia	Cameroon	Democratic Republic of the Congo	Democratic Republic of the Congo	Democratic Republic of the Congo	United Kingdom	Netherland	Florida
Smallpox vaccination history	None	None	None	None	None	None	None	None	None	None	None	None	None	None	None	None	None
Chickenpox vaccination history	None	None	None	None	None	None	None	None	None	None	Yes	None	None	None	None	Yes	None
HIV, hepatitis B, and hepatitis C status	None	None	None	None	Negative	Negative	None	None	None	None	Negative	None	None	None	None	Negative	Negative
Time to qPCR negativity, days after fever onset (days)	-	-	-	-	-	-	-	-	-	-	-	-	-	-	19	-	-
Prodrome (days)	2-3	4	5	-	5	3	2	3	2	9	1	-	-	-	-	-	5
Lymphade-nopathy	Yes	No	Yes	No	No	No	No	No	No	Yes	Yes	No	No	No	Yes	No	No
Approximate maximum number of concurrent lesions	-	-	>250	-	-	-	-		-	-		-	-	-	30	20	-
Distribution of lesions	Mouth, neck	-	Face, mouth, oropharynx, chest, upper and lower extremities and the palms and soles	Face, mouth, oral mucosa, trunk, back, palms, and genital area	Palms of the hands and sole of the feet	Palms of the hands and soles of the feet	-	Palms, foot soles, and mucous membranes	Face, mouth, arms, trunk, and legs	Trunk, face, palms, genitals and soles of the feet	Face, chest, arms and legs, including his soles and palms	Head, palms of the hands, foot	-	-	Face, trunk, arms, and legs	Left ear, left lower jaw, both forearms, and both thighs and on the back	Arms, legs, and trunk
Complications of illness	Disseminated rash	Fever, polyadenopathy, facial edema, severe erosive pharyngitis, hepatosplenomegaly, diarrhea, vomiting, and a few varicella-like skin eruptions	Swollen, painful cervical lymph nodes, dysphagia, vomiting, difficulty breathing, and an inability to eat or drink.	Sweats, chills, vomiting, loss of appetite, cough, and pruritus	Facial edema, bilateral conjunctivitis, pulmonary edema	Fever and headaches	Fever and a few pruritic vesicles	Stomatitis, rhinitis, conjunctivitis, cough, severe left-sided cervical lymphadenitis	Skin rashes, fever, weakness, and severe body pain	Fever, extensive generalized papular rash, headache, malaise, sore throat, oral and nasal mucosal lesions, and ulcers	Superadded bacterial skin and bilateral conjunctival injection	Fever, Skin eruption, pruritus	Fever	Fever, Skin eruption, Pruritus, Abdominal pain	Pruritis and contact dermatitis from cleaning products	Dermatomycosis, impetigo vulgaris	Molluscum contagiosum
Specific management of complications	-	Antibiotic and quinine therapy	(Day 1) intravenous diphenhydramine, lorazepam, and morphine; (Day 2) intravenous ampicillin/sulbactam, 200 mg/kg/day divided every 6 h for the retropharyngeal phlegmon; (Day 4) Bacitracin cream was applied to the lesions on her face to ameliorate scarring.		intravenous antibiotics and tetracycline eye ointment; treated with furosemide and oxygen, and profound hypothermia	Oral antibiotics	Promethazine	intravenous amoxicillin-clavulanic acid, retinol tablets, antibiotic eye drops, paracetamol, diluted plumpy nut, and intravenous maintenance fluids; (Day 2-5) i.v. ceftriaxone, and pain management was intensified to include morphine.	Analgesics and antibiotics	Antibiotics, antipyretics, and topical medication	(Initial) calamine lotion and paracetamol; (confirmation) oral cloxacillin 500 mg four times daily for 7 days and tetracycline 1% eye ointment for 5 days	Symptomatic treatment	Symptomatic treatment	Symptomatic treatment	Calamine lotion and a short course of antibiotics at the onset of dermatitis	Antifungal cream and antibiotic cream	intravenous antibiotics, Prophylactic trifluridine drops
Blood	Yes	Yes	Yes	Yes	Yes	Yes	No	Yes	Yes	Yes	Yes	No	No	No	Yes	Yes	Yes
Nose or throat	No	-	-	Yes	No	No	No	No	Yes	No	Yes	No	No	No	Yes	Yes	Yes
Urine	No	-	Yes	-	No	No	No	No	No	No	No	No	No	No	No	Yes	No
Laboratory analysis	-	Increased lymphoid cells; plasmodium falciparum detected	Peripheral white Blood Cells - 17 900 cells/mm^3^; protein: 5.7 g/dl; albumin: 2.3 g/dl	Positive for the presence of Orthopoxvirus immunoglobulin G and immunoglobulin M	-	-	-	Negative for measles	-	-	-	-	-	-		immunoglobulin A deficient: 0.45 g/L; normal erythrocyte sedimentation rate (12 mm/h; reference range: 0–13 mm/h) and a low C-reactive protein concentration (1.9 mg/L; reference range: 0–5 mg/L)	-
Antivirals received	No	No	No	-	No	No	No	No	-	Yes	No	No	No	No	No	No	tecovirimat and Vaccinia Immune Globulin Intravenous
Day of illness treatment commenced	-	4	5	2	3	11	1	3	2	9	2	-	-	-	-	16	5
Complications of treatment	-	-	-	-	Oral and genital lesions and the pruritus got worse on promethazine	-	Agitation and hypotonia	-	-	-	-	-	-	-	-	-	Lesions subsequently spread to the back, soles of feet, face, and eyelid and became pustular
Duration of hospitalisation with MPV, days	1	2	7	0	8	33	3	12	-	23	7	14	14	14	22	0	10
Biopsy	Yes	No	No		No		No	-	No	No	No	No	No	No	No	No	No
Outcome of MPV infection	Died	Died	Full recovery	Full recovery	Died	Partial resolution	Died	Died	Full recovery	Full recovery	Full recovery	Full recovery	Full recovery	Full recovery	Full recovery	Partial resolution	Full recovery
Type of study	Case study	Case study	Case study	Case study	Case study	Case study	Case study	Case study	Case study	Case study	Case study	Case study	Case study	Case study	A retrospective observational study	Case study	Case study

**Table 3:** Analysis of the clinical progression and therapeutic response of monkeypox virus in pregnant women MPV: Monkeypox virus

Patient number	18 [17]	19 [17]	20 [17]	21 [17]
Year of infection	March 2007 to July 2011			
Age	20	25	29	22
Time of gestation, weeks	6	6–7	14	18
Country of acquisition	Democratic Republic of the Congo	Democratic Republic of the Congo	Democratic Republic of the Congo	Democratic Republic of the Congo
Smallpox vaccination History	None	None	None	None
HIV, hepatitis B, and hepatitis C, Malaria status	Malaria: negative	Malaria: negative	Malaria: negative	Malaria: positive
Prodrome	-	-	-	-
Lymphadenopathy	-	-	-	-
Approximate maximum number of concurrent lesions	76	1335	16	113
MPV load, genome copies/mL				
Maximum	3.5 × 10^3^	7.9 × 10^5^	2.3 × 10^5^	8.9 × 10^5^
In placental tissue	-	-	-	2.4 × 10^7^
In fetal tissue	-	-	-	1.6 × 10^3^
Distribution of lesions on mother	-	-	-	-
Distribution of lesions on fetus	-	-	-	Head; the trunk, including the abdomen, back, and chest; and the extremities, including the palms and soles of the hands and feet
Specific management of complications	Analgesics (paracetamol and papaverine), antibiotics (amoxicillin, chloramphenicol through eye drops, erythromycin, and gentamycin, if required), and worm medications (metronidazole and mebendazole) were administered.	Analgesics (paracetamol and papaverine), antibiotics (amoxicillin, chloramphenicol through eye drops, erythromycin, and gentamycin, if required), and worm medications (metronidazole and mebendazole) were administered.	Analgesics (paracetamol and papaverine), antibiotics (amoxicillin, chloramphenicol through eye drops, erythromycin, and gentamycin, if required), and worm medications (metronidazole and mebendazole) were administered.	Analgesics (paracetamol and papaverine), antibiotics (amoxicillin, chloramphenicol through eye drops, erythromycin, and gentamycin, if required), and worm medications (metronidazole and mebendazole) were administered; quinine for malaria.
MPV DNA detected				
Blood	Yes	Yes	Yes	Yes
Nose or throat	No	No	No	No
Urine	Yes	Yes	Yes	Yes
Antivirals received	No	No	No	No
Disease onset to outcome (days)	24	14	9	21
Day of illness treatment commenced	-	-	-	-
Complications of Treatment	-	-	-	-
Time to qPCR negativity, d after fever onset	26	>17	2	>27
Minimum albumin level, g/dL	2.6	2.4	2.4	1.8
Outcome of monkeypox virus Infection	Miscarriage	Miscarriage	Live birth	Fetal death
Type of study	An observational study	An observational study	An observational study	An observational study

Discussion

MPV is a self-limiting double-stranded DNA virus. Children, pregnant women, and immunocompromised people may have serious conditions. Children's case fatality rate is 0-11%. MPV was initially found in a nine-month-old newborn who had not been vaccinated against smallpox in 1970. All 63 African children death in the 1970s-1990s were under 10 years. Just 37.5% of children in the same age group died from 2000 to 2019. In 2014 and 2016, all suspected MPV cases in the DRC were in males under 15 years, with 57.8% among 15-18-year-olds. Sixty percent of Republic of the Congo infected were under 15 years [27]. Epidemiological information from earlier MPV outbreaks in Africa suggests that smallpox-unvaccinated household contacts of MPV-infected patients may have a subsequent attack incidence of 123%, particularly among minors under 15 years [28]. Mother-to-child transmission or nosocomial infection in hospitals is rare. Some clinical data suggest first-trimester sickness may cause miscarriages [17]. In 2003, MPV was first found in children and adults in the US when prairie dogs were kept with ill Gambian giant rats from Ghana [29]. Early symptoms include rash, fever, chills, and lymphadenopathy. Lesions on the palms, soles, and mucosal membranes are uncommon. Children typically develop lesions on the face, torso, and upper extremities with a linear pattern, suggesting autoinoculation of the virus through scratching [30].

MPV prevention and treatment initiatives for children and pregnant women

Currently, there is no vaccine authorized for use against MPV. Observational studies have shown that smallpox immunizations provide up to 85% protection against MPV. Eliminating smallpox immunization will make more people susceptible to MPV. The CDC recommends brincidofovir, tecovirimat, cidofovir, or vaccinia immune globulin for severe cases, children, and persons with compromised immune systems [31]. Tecovirimat (TPOXX®/ST-246), which inhibited Orthopoxvirus VP37 envelope-wrapping protein and was FDA-approved in 2018, is indicated against smallpox infection caused by the Variola virus in adults and children [32]. It is available in 200mg capsules or intravenously. Intravenous tecovirimat is contraindicated for severe renal impairment. This group can take oral formulations. Intravenous tecovirimat should be used cautiously in patients with moderate or mild renal impairment and children under two years old due to undeveloped renal tubular function [33]. The FDA authorized brincidofovir on 4 June 2021 to treat human smallpox in adults, children, and infants. MPV treatment with brincidofovir is unknown. Its anti-orthopoxvirus activity has been shown in animals and in vitro [33].

Probenecid should be used with care in children, pregnant women, and those who are allergic to sulfa drugs [34]. Among the second and third-generation vaccines, LC16 and MVA have been approved for use in children in Japan and the United States, respectively [35]. For pre-and postexposure prophylaxis during pregnancy, the non-replicating smallpox vaccine (MVA-BN) is suggested [36]. The same non-replicating MVA viral vector serves as the basis for various Ebola virus illnesses (EVD), including MVAfilo (marketed as Mvabea™). The European Union has licenced this EVD vaccination for adults and children older than one year. A vaccine against respiratory syncytial virus infection is also being developed using the MVA viral vector technology. A total of nine studies corroborate the product’s favorable safety profile when employing for the prevention of EVD, and some data suggest that operating as a vector does not influence the immune response to MVA. In addition, there is no indication of prenatal damage in animal models. Allergy patients should take the MVA-BN vaccination with care. Healthcare practitioners and vaccination managers must be prepared for MVA-BN-induced anaphylaxis. Injection site responses (itching, induration, swelling, redness, pain) and systemic reactions such as muscular discomfort, headache, myalgia, nausea, tiredness, and chills were the most prevalent adverse effects of MVA-BN (more than one in 10 vaccine recipients). Atopic dermatitis may intensify or flare up, causing more extreme local skin responses like itching, swelling, and redness, and additional general symptoms including headache, muscular discomfort, and feeling ill or exhausted [35].

There are little data on the safety of ACAM2000 or LC16 in pregnant women and children. Warnings and precautions apply to PLWH, children, and pregnant women, where ACAM2000 may damage fetuses. Lactating mothers may accidentally inoculate their infants with ACAM2000 live vaccinia virus, causing difficulties. Inoculation site responses, lymphadenitis, and constitutional symptoms, including myalgia, fever, tiredness, malaise, and headache, are common ACAM2000 side effects. ACAM2000 may Stevens-Johnson syndrome, erythema multiforme, and skin infections. Myocarditis, pericarditis, post-vaccinal encephalitis, and encephalopathy have been documented [35]. The Global Advisory Committee on Vaccine Safety (GACVS) advised that the use of smallpox vaccinations be governed by the predicted risk vs. benefit during a different epidemic or exposure scenarios. This evidence must be evaluated within the context of MPV [35]. The characteristics and potential adverse effects of children’s vaccinations for the management of MPV are listed in Table 4.

**Table 4:** Characteristics of vaccines prepared for children

Vaccine	Characteristics of vaccine	Potential adverse events
First generation of smallpox vaccine (e.g., Dryvax, EM63, Tiantan/Temple of Heaven, Lister, and Aventis Pasteur Smallpox Vaccine, among others)	Several different vaccinia virus strains were employed in vaccines administered throughout the eradication campaign. Almost all were derived from calf lymph. All vaccinations of the first generation included live replication-capable viruses.	Postvaccination encephalitis is an uncommon but severe adverse effect, especially in children less than two years old [37].
Second generation of smallpox vaccine (e.g., ACAM2000, CJ-50300, VV Lister/CEP, Elstree-BN, and Lister vaccine produced in primary rabbit kidney cells (RIVM))	Vaccines of the second generation are generated using tissue cell culture and appropriate manufacturing standards. As a result, they are less likely to be contaminated by accidental substances. As both first- and second-generation vaccinations include live, replication-competent vaccinia virus, they are expected to have similar side effects.	Postvaccination encephalitis is an uncommon but severe adverse effect, especially in children less than two years old [37].
Third-generation MVA-BN (modified vaccinia Ankara-Bavarian Nordic)	This is available in a liquid frozen formulation intended to be two dosages given four weeks apart. The United States has given emergency authorization for usage in patients under the age of 18 years [35].	-
Third-generation LC16 (KM Biologics)	Single dosage. Approved for use in newborns, children, and adults of all ages in the USA [35].	-

A viral swab is tested for MPV using PCR, which may differ between MPV and other orthopoxviruses. There is currently no accepted MPV test; instead, positive results are often verified by national reference labs [38]. Roche (Basel, Switzerland), a pharmaceutical company, stated on 25 May 2022 that they had created a detection kit for MPV using quantitative PCR. Swabs from open sores or vesicles are put in a vial of viral culture media or viral transport medium to send to a virology lab. If all lesions have crusted, scrape swabs into a dry, basic, universal container. An EDTA blood sample and throat swab should also be taken if the patient exhibits systemic symptoms including a fever, rash, or sore throat. High-risk contacts of confirmed cases must have systemic symptoms but no rash or lesions to give samples [38]. Given the short period of viremia, swabs, swab samples, and aspirated lesion fluid should be prioritized above blood samples if lesions are present.

The danger to the fetus is still unquantifiable due to a lack of evidence on MPV during pregnancy; nonetheless, it indicates that vertical transmission and fetal death are feasible. As a result, pregnant women with a confirmed MPV should proceed with caution until further evidence becomes available. If the pregnancy is less than 26 weeks long or if the mother is ill, cardiotocography should be used often (2-3 times daily) to check on the health of the fetus. The health of the baby and the placenta should be monitored routinely through ultrasound during the acute infection. This would be done during the first trimester to check viability and provide screening. Second-trimester evaluations should involve a comprehensive anatomy scan, a measurement of amniotic fluid volume, and two sets of fetal biometry spaced 10-14 days apart. Ten to fourteen-day intervals of fetal biometry, a comprehensive anatomy scan, a measurement of amniotic fluid volume, and fetal Doppler are all appropriate for evaluation in the third trimester. It is believed that the danger to the baby is low after the maternal infection has cleared up; nonetheless, given data are few, it is prudent to consider continuing to monitor the fetus with scans every four weeks throughout the remainder of the pregnancy.

Even though the present epidemic has been traced to the west African lineage of the MPV, most cases are mild and self-limiting. Considering gestational age, fetal state, and Caesarean conditions, the baby should be delivered if there is fetal compromise or the mother's life is in risk. The unit policy calls for magnesium sulfate to be given to premature infants to preserve their developing brains. Using steroids to help the fetus develop in case of preterm delivery is not anticipated to have a serious negative impact on the health of the mother. Nonetheless, its intended usage has to be reviewed with the virologist and the woman’s larger multidisciplinary care team.

In a woman with an active MPV, there is no evidence to suggest a particular method of delivery is preferable. Because of the high probability of vertical transmission, the infant may be infected before delivery, making a caesarean section unnecessary. Contact with open MPV lesions is known to spread the virus. Hence, genital lesions might cause neonatal infections during labor and delivery. If genital lesions are discovered, a caesarean section is suggested since newborns have the greatest chance of severe MPV. After considering the (unquantifiable) risk of neonatal infection, a woman with verified or assumed MPV should have a caesarean section. Transplacental transfer of maternal IgG antibodies is expected to begin seven days after rash development, which protects the newborn; hence in most situations, it is not suggested that infected people undergo delivery shortly [36]. If a patient’s vaginal and rectal PCR tests are negative, they may be able to give delivery vaginally. In order to protect the newborn from catching an infection from the mother’s sores or exudates, specialists advise having a caesarean section instead of a vaginal delivery. If there are lesions in the oropharynx, general anesthesia may be complicated, whereas lesions in the skin close to the insertion site may need neuraxial anesthesia [39].

Newborn care is determined by the manner of birth and the likelihood of vertical MPV transfer. Babies should be checked for irritability, feeding issues, and any signs of skin, eye, or mucous membrane lesions. Babies delivered through caesarean section may not need therapy, but those at high risk for MPV transmission after a vaginal delivery should undergo PCR testing using skin, oropharynx, and rectal swabs and perhaps get treatment with vaccinia immune globulin. Patients at low risk should wait to breastfeed or engage in skin-to-skin contact until isolation is complete. Breastfeeding may be an option for high-risk newborns with a positive PCR if there are no lesions present on the breast [36]. The primary method used to avert the spread of MPV is to inform the public about the dangers the disease poses and how they may lessen their chances of contracting it. Research on the effectiveness and safety of vaccination as a means of MPV control and prevention is now underway. Several nations already have or are formulating plans to vaccinate employees in potentially hazardous environments, such as hospitals, laboratories, and emergency response teams.

Rapid case detection and surveillance are essential for stopping an epidemic in its tracks. MPV transmission during human pandemics is most likely via contact with infected persons. Healthcare workers and the public have greater infection rates. Healthcare practitioners should adopt routine infection control practices when caring for patients with suspected or confirmed MPV or while handling specimens from these patients. Wherever possible, healthcare providers should be selected from among those who have had the smallpox vaccination. Trained personnel using appropriately equipped labs should handle samples collected from humans and animals suspected of having MPV. The WHO recommends using triple packing for transporting infectious material, including patient specimens. To prevent the spread of MPV, any animals that have come into touch with an infected one must be isolated for 30 days, treated with care, and monitored for the disease. Table 5 offers an overview of some regional and national norms and policies adopted for the prevention of MPV throughout the globe [40].

**Table 5:** An overview of some regional and national norms and policies adopted for the prevention of MPV throughout the globe MPV: Monkeypox virus; WHO: World Health Organisation; ACIP: Advisory Committee on Immunization Practices

	Guideline	Overview
WHO [41-46]	WHO: Clinical management and infection prevention and control for monkeypox – Interim rapid response guidance (2022)	These are MPV treatment and infection prevention recommendations for hospital and community settings. The recommendations include post-infection care, including medication, diet, and psychological aid.
	WHO: Laboratory testing for the monkeypox virus – Interim guidance (2022)	The overarching purpose of laboratory testing here is to provide rapid and reliable confirmation of infection to back up breaking chains of transmission and therefore put a halt to the epidemic.
	WHO: Public health advice for gatherings during the current monkeypox outbreak (2022)	This publication is intended to serve as a public health resource for local governments, public health authorities, national or international organizers, and professional staff engaged in the planning and implementation of meetings of any size or scope.
	WHO: Risk communication and community engagement (RCCE) for monkeypox outbreaks – Interim guidance (2022)	It lays forth suggestions, factors to consider, and approaches to help individuals at risk make educated choices to protect themselves and others from MPV. Tips for reaching out to impacted communities and other crucial audiences while preventing the spread of stigmatizing messages are provided.
	WHO: Surveillance, case investigation, and contact tracing for mpox (monkeypox) – Interim guidance (2022)	The MPV has been consistently renamed to mpox throughout the document in accordance with the latest WHO guidelines. Furthermore discussed are the potential uses of wastewater monitoring in detecting mpox transmission in communities and a more in-depth account of the inquiry into suspected animal exposure.
	WHO: Vaccines and immunization for monkeypox – Interim guidance (2022)	In this interim guideline, the WHO offers vaccination and prevention advice for MPV.
Canada [47-50]	National Advisory Committee (NACI): Rapid response on interim guidance on the use of Imvamune in the context of monkeypox outbreaks in Canada (2022)	Independent advice and suggestions based on state of the art in science are included in this statement.
	Public Health Agency Canada (PHAC): Canadian Immunization Guide - Smallpox and monkeypox vaccine (2014, updated 2022)	If an outbreak of smallpox or MPV were to occur in Canada or anywhere else, these measures would be recommended to be performed.
	PHAC: Interim guidance on infection prevention and control for the suspect, probable, or confirmed monkeypox within healthcare settings (2022)	This may help in determining the extent to which healthcare workers are exposed to MPV in the workplace.
	PHAC: Monkeypox – Public health management of cases and contacts in Canada (2022)	In the event that the MPV is suspected or confirmed within their jurisdictions, this document provides instructions to PHAs operating at the federal, provincial, and territorial (FPT) levels.
United States [51-56]	Advisory Committee on Immunization Practices (ACIP): Use of JYNNEOS (smallpox and monkeypox vaccine, live, non-replicating) for preexposure vaccination of persons at risk for occupational exposure to orthopoxviruses – Recommendations, United States (2022)	This should be taken into account while selecting between JYNNEOS and ACAM2000 as the main vaccine.
	American Society of Anesthesiologists (ASA)/Anesthesia Patient Safety Foundation (APSF): Statement on monkeypox (2022)	The statement is meant to educate those working in the field of anesthesia about MPV.
	CDC: Considerations for reducing mpox transmission in congregate living settings (2022)	These provide factors to think about in limiting the spread of mpox in communal living situations.
	CDC: Interim clinical considerations for use of JYNNEOS and ACAM2000 vaccines during the 2022 US mpox outbreak (2022)	As the 2022 mpox epidemic in the United States approaches, researchers explore interim clinical considerations for using the JYNNEOS and ACAM2000 vaccines.
	CDC: Interim guidance for prevention and treatment of monkeypox in persons with HIV infection, United States (2022)	Temporary recommendations for the treatment and prevention of MPV in HIV-infected people are included in this document.
	CDC: Mpox – Information for healthcare professionals	Information for medical experts is included in this document.
Europe [57-61]	European Centre for Disease Prevention and Control (ECDC): Considerations for contact tracing during the monkeypox outbreak in Europe (2022)	Stochastic simulations of MPV epidemics are presented in this research using a unique mathematical model. Together with metrics for public health authorities in the EU/EEA to utilize in gauging the success of their contact tracing efforts, this report provides guidelines for the prioritization of efforts to identify and manage close relationships.
	ECDC: Interim advice for public health authorities on summer events during the monkeypox outbreak in Europe (2022)	With the help of this document, public health officials will be able to reduce the potential threat that MPV poses to the public by effectively distributing accurate information, expert advice, and actionable direction to participants.
	ECDC: Interim advice on risk communication and community engagement during the monkeypox outbreak in Europe (2022)	In light of the recent MPV epidemic in Europe, this material is meant for health authorities working on RCCE. Based on the epidemiology and context of the epidemic, the suggested preventative actions, and people’s views and behaviour, it offers advice on ways to communicate risks and participation of demographic groups.
	ECDC: Risk assessment – Monkeypox multi-country outbreak (2022)	The global outbreak of MPV risk assessment is the subject of this report.
	ECDC: Risk communication and community engagement approaches during the monkeypox outbreak in Europe (2022)	Health authorities are encouraged to use this document as a guide for formulating RCCE actions in response to the ongoing MPV epidemic in Europe.
United Kingdom [62-64]	British HIV Association (BHIVA): Rapid statement on monkeypox virus (2022)	This consists of prompt MPV guidance.
	UK Health Security Agency (UKHSA): Mpox (monkeypox) – Guidance (2022)	Guidelines for healthcare practitioners, recommendations for immunization, recommendations for the general public, and a technical and epidemiological overview and monitoring and surveillance system are all included.
	UK Health Security Agency (UKHSA): The Green Book – Smallpox and monkeypox (2013, updated 2022)	Vaccination information against communicable diseases such as smallpox and MPV is included.
Australia and New Zealand [65-68]	Australian Technical Advisory Group on Immunisation (ATAGI): Clinical guidance on vaccination against monkeypox (2022)	Advice about getting the smallpox vaccination to avoid getting the MPV virus.
	Communicable Diseases Network Australia (CDNA): National guidelines for public health units on monkeypox virus infection (2022)	The recommended public health measures for cases and contacts of MPV virus infection are outlined in these interim recommendations.
	Infection Prevention and Control Expert Group (ICEG): Interim guidance on monkeypox for health workers (2022)	This includes recommendations for medical personnel on MPV.
	Public Health Laboratory Network (PHLN): Guidance on monkeypox patient referral, specimen collection and test requesting for general practitioners and sexual health physicians (2022)	This document includes guidelines for sending people suspected of having MPV to primary care and sexual health providers. Instructions for collecting and transporting specimens in a secure manner are also included.

It would be unreasonable to interpret our results without considering the following limitations, despite the fact that we made considerable precautions to minimize any bias and decrease the heterogeneity at every stage. In the case studies, we were unable to determine the mean or standard deviation. Several of the research studies have a lot of discrepancies among them. Few studies have looked at how vertical transmission of MPV from mother to child affects pregnancy outcomes during outbreaks of the disease.

## Conclusions

It is unfortunate that vaccination adoption is still a problem. Health systems must immediately begin preparing and educating communities with clear, basic, and truthful information in order to safeguard vulnerable populations, including pregnant women, children, and others. Public health measures should be broadly adopted to safeguard vulnerable groups, particularly those who are immunocompromised, pregnant women, and children. Obstetricians should always be ready to treat a patient who is pregnant. The difficulty of clinical diagnosis and treatment is compounded by the fact that some patients exhibit no symptoms at all. Also, further study into MPV’s impact on expecting mothers is required. Findings suggest a lack of diagnostic equipment in rural health centers as well as expert health workers to recognize the disease. Also, practical hurdles, such as a lack of knowledge on collecting and transferring a sample and staff nervousness about handling infected material, have been seen in other countries and slowed down the diagnosis process.

By doing this comprehensive analysis, we want to alert medical professionals to the fact that MPV may emerge in young people and is widespread. In cases where clinical signs may be connected to MPV, we recommend rapid diagnostic testing to avoid the spread of the virus in the community. We recommend immunization for high-risk contacts as a means of stopping the spread of illness.
